This article has been retracted.

# Effect of Vitamin D Combined with Recombinant Human Growth Hormone in Children with Growth Hormone Deficiency

**DOI:** 10.1155/2022/7461958

**Published:** 2022-07-19

**Authors:** Pingping Wang, Xuefeng Jin, Yan Zhang, Jianmei Zhang, Yunfang Li, Suhong Yang, Dan Li

**Affiliations:** ^1^Department of Endocrinology, Hangzhou Children's Hospital, No. 195 Wenhui Road, Gongshu District, Hangzhou, Zhejiang 310014, China; ^2^Department of Gastroenterology, Hangzhou Children's Hospital, No. 195 Wenhui Road, Gongshu District, Hangzhou, Zhejiang 310014, China; ^3^Hangzhou D.A. Medical Laboratory, Building 1, 329 Jinpeng Street, Sandun Town, Xihu District, Hangzhou, Zhejiang 310012, China

## Abstract

**Objective:**

Growth hormone deficiency (GHD) refers to the complete or partial lack of pituitary growth hormone synthesis and secretion. This study is aimed at investigating the efficacy of vitamin D and recombinant human growth hormone (rhGH) in children with GHD.

**Methods:**

A total of 100 children with GHD at our hospital were included between 1^st^ January 2018 and 31^st^ October 2020. The patients were divided into a study group (*n* = 70, received vitamin D combined with rhGH) and a control group (*n* = 30, received rhGH). The growth and development (bone age, growth rate, and height), bone metabolism (bone alkaline phosphatase (BAP), *β*-collagen degradation product (*β*-CTX), osteocalcin (OC), and amino-terminal propeptide type I procollagen (PINP)), insulin-like growth factor 1 (IGF-1), ghrelin, and adverse reactions in the two groups were measured before and 12 months after treatment.

**Results:**

There were no significant differences in the bone age, growth rate, and height between the two groups before treatment. After 12 months of treatment, the bone age, growth rate, and height of the study group were significantly higher than those of the control group. After 12 months of treatment, the levels of serum BAP, PINP, and OC in the study group were significantly higher than those in the control group, while the levels of *β*-CTX in the study group were significantly lower than those in the control group. The serum IGF-1 level in the study group was significantly higher than that in the control group, while the ghrelin level in the study group was lower. There was no significant difference in the incidence of adverse reactions between the two groups.

**Conclusion:**

Combined rhGH and vitamin D treatment can promote growth and development, improve bone metabolism, and regulate IGF-1 and ghrelin levels.

## 1. Introduction

Growth hormone deficiency (GHD) is characterized by the complete or partial deficiency of pituitary synthesis and secretion of the growth hormone or growth and developmental disorders caused by receptor defects and structural abnormalities [1–3]. GHD is an important cause of slow growth and short stature in children. Affected children may have short stature, growth retardation, dyslipidemia, and other nutritional disorders. Some patients also have neurological abnormalities that pose a major threat to the patient's physical and mental health, growth, and development [4–6]. Therefore, effective measures should be taken to treat children with GHD.

Recombinant human growth hormone (rhGH) is an important drug for the treatment of GHD. It can promote the regulation of the endocrine system and muscle and bone growth, as well as protein synthesis, thus playing a therapeutic role in GHD [7]. However, it is difficult to achieve optimal results with rhGH alone. Clinical studies have shown that vitamin D can affect calcium metabolism, maintain body growth and development, and promote osteoblast proliferation and bone matrix formation. However, vitamin D expression is low in children with GHD; therefore, vitamin D supplementation is of great significance in promoting the growth and development of children with GHD [8].

The purpose of this study was to investigate the clinical application effect of vitamin D and rhGH on the treatment of GHD.

## 2. Methods

### 2.1. Patients

The children with GHD treated in our hospital from 1^st^ January 2018 to 31^st^ October 2020 were enrolled in this study. Participants signed informed consent, and the study protocol was approved by the Ethics Committee of Hangzhou Children's Hospital.

The inclusion criteria for this study were (1) growth velocity < 5 cm/year; (2) delayed bone age; (3) growth hormone release test, peak growth hormone < 10 *μ*g/L; (4) normal mental development; (5) age ≤ 12 years; and (6) no abnormality found in chromosome examination. Exclusion criteria are (1) patients with chromosomal or genetic metabolic diseases, (2) patients with abnormal thyroid function, (3) patients who have received vitamin D treatment within 3 months before the study, (4) patients with mental disorders, (5) allergies, (6) congenital malformations, and (7) those with dysfunction of kidneys, livers, and other organs.

### 2.2. Intervention

The patients in both groups were treated with routine interventions (such as nutrition supplements and developing daily routines) and growth exercises. Regarding the growth exercise for increasing the height, patients were instructed to exercise for 30 minutes before going to bed every night, 15 minutes/time, and perform 300 to 500 hops a day and jumping, stretching, and other whole-body exercises for 30 minutes. Furthermore, rhGH (Changchun GeneScience Pharmaceuticals Co. Ltd, CFDA No. S20050024) was injected subcutaneously at 0.12 IU/(kg·d) every night before going to bed in the control group. The patients in the study group received vitamin D_3_ drops (Sinopharm Xingsha Pharmaceutical Co., LTD. (Xiamen), SFDA approval number H35021450), 400 IU once a day. Both groups were treated for 12 months.

### 2.3. Observation Indexes

The growth status of the two groups of patients before and 12 months after treatment, including bone age, growth rate, and height, was analyzed. The bone metabolism of the two groups before and 12 months after treatment was statistically analyzed. Blood samples were collected from each patient. Electrochemical fluorescence immunoassay was used to detect bone-specific alkaline phosphatase (BAP), *β*-collagen degradation product (*β*-CTX), and amino-terminal propeptide type I procollagen (PINP), and the enzyme-linked immunosorbent assay was used to detect osteocalcin (OC), insulin-like growth factor-1 (IGF-1), and growth hormone (ghrelin) levels (ProteinTech, China). The adverse reactions of the two groups of patients were determined.

### 2.4. Statistical Analysis

The data analysis was performed using SPSS22.0 software (IBM SPSS Statistics, Chicago, USA). The measurement data were expressed as the mean ± *s*, and the *t*-test was used for comparison of differences between the two groups. The enumeration data were expressed as *n* (%), and *χ*^2^ was used as the test for comparison. Two-sided *P* value less than 0.05 was considered a significant difference.

## 3. Results

### 3.1. Baseline Data

A total of 102 children with GHD in our hospital from 1^st^ January 2018 to 31^st^ October 2020 were selected. However, two patients who have received vitamin D treatment within 3 months before the study were excluded. The patients were divided into the study group (*n* = 70, taking vitamin D combined with rhGH) and the control group (*n* = 30, taking rhGH alone) according to the treatment schedule. There were 37 boys and 33 girls in the study group. The average age was 7.51 ± 2.39 years, ranging from 4 to 12 years. The height ranged from 90.3 to 131.9 cm, with an average of 101.76 ± 22.19 cm; the growth rate ranged from 3.2 to 4.8 cm/year, with an average of 4.01 ± 0.35 cm/year. Bone age ranged from 2 to 9 years, with an average of 5.69 ± 1.91 years. In the control group, there were 16 boys and 14 girls; the average age was 7.23 ± 2.51 years, ranging from 4 to 12 years. The height ranged from 89.5 to 133.7 cm, with an average of 103.11 ± 20.69 cm. The growth rate ranged from 3.1 to 4.9 cm/year, with an average of 3.98 ± 0.38 cm/year. The clinical parameters of sex, age, height, growth rate, and bone age were comparable between the two groups (*P* > 0.05).

### 3.2. Comparison of Growth and Development between the Two Groups

There were no significant differences in the bone age, growth rate, and height between the study group (5.69 ± 1.91 years, 4.01 ± 0.35 cm/year, and 101.76 ± 22.19 cm, respectively) and the control group (6.02 ± 2.04 years, 3.98 ± 0.38 cm/year, and 103.11 ± 20.69 cm, respectively) before treatment (*P* > 0.05). After 12 months of treatment, the bone age, growth rate, and height of the study group (9.01 ± 1.10 years, 9.62 ± 2.38 cm/year, and 139.81 ± 16.53 cm, respectively) were higher than those of the control group (9.03 ± 0.98 years, 7.91 ± 2.11 cm/year, and 128.64 ± 13.79 cm, respectively) (*P* < 0.05; Table 1).

### 3.3. Comparison of Bone Metabolism between the Two Groups

There were no significant differences in the serum levels of BAP, *β*-CTX, OC, and PINP between the study group (89.67 ± 26.12 U/L, 0.83 ± 0.29 *μ*g/L, 59.79 ± 17.10 *μ*g/L, and 469.62 ± 97.73 *μ*g/L, respectively) and the control group (91.23 ± 28.09 U/L, 0.87 ± 0.35 *μ*g/L, 61.56 ± 15.53 *μ*g/L, and 473.68 ± 93.56 *μ*g/L, respectively) before treatment (*P* > 0.05). After 12 months of treatment, the levels of serum BAP, PINP, and OC in the study group (173.64 ± 44.69 U/L, 589.97 ± 103.13 *μ*g/L, and 83.37 ± 15.32 *μ*g/L, respectively) were higher than those in the control group (132.12 ± 39.64 U/L, 541.66 ± 94.92 *μ*g/L, and 74.29 ± 12.37 *μ*g/L, respectively), while the levels of *β*-CTX of the study group (0.42 ± 0.18 *μ*g/L) were lower than those in the control group (0.59 ± 0.20 *μ*g/L) (*P* < 0.05), as shown in Table 2.

### 3.4. Comparison of IGF-1 and Ghrelin Levels between the Two Groups

There was no significant difference in the serum levels of ghrelin and IGF-1 between the study group (6.89 ± 0.94 ng/mL and 98.29 ± 13.19 ng/mL, respectively) and the control group (7.01 ± 1.10 ng/mL and 102.68 ± 15.64 ng/mL, respectively), before treatment (*P* > 0.05). After 12 months of treatment, the serum IGF-1 level in the study group (173.05 ± 19.37 ng/mL) was higher than that in the control group (151.36 ± 16.62 ng/mL), whereas the ghrelin level of the study group (4.56 ± 0.39 ng/mL) was lower than that in the control group (5.38 ± 0.46 ng/mL) (*P* < 0.05; Table 3).

### 3.5. Comparison of Adverse Reactions between the Two Groups

As shown in Table 4, there was no significant difference in the incidence of adverse reactions between the study group (2.86%) and the control group (9.99%) (*P* > 0.05).

## 4. Discussion

GHD is mainly caused by the insufficient secretion of the growth hormone from the anterior pituitary. It is an important cause of short stature in children. Studies have shown that GHD can result in low bone age/actual age, slow bone maturation, slow growth rate, and short stature in children as well as systemic organ system and metabolic disorders, which pose a great threat to the physical and mental health of children and their parents [9–11].

rhGH is an important drug for the clinical treatment of GHD. It can prevent growth disorders caused by the insufficient secretion of the growth hormone in addition to downregulating the sensitivity of peripheral tissues to insulin, effectively maintaining the nutrient supply of the body, and providing nutrients for the growth and development of children with GHD. It can also promote the body's metabolism to improve body function [12–14]. In addition, research indicates that vitamin D can promote the absorption of phosphorus, calcium, and other substances, accelerate bone growth, and improve bone development. As it is an important factor that promotes bone growth and development, vitamin D can also be combined with rhGH for treating GHD [15, 16]. In this study, rhGH and vitamin D were combined to treat children with GHD in our hospital. It was found that the, growth rate, and height of the study group were higher than those of the control group, and the improvement in bone metabolism-related indices (BAP, *β*-CTX, OC, and PINP) was significantly greater than that in the control group, indicating that combined rhGH and vitamin D has high application value in GHD. The combination can improve bone metabolism and promote growth and development in children. This is because the occurrence and progression of GHD are closely related to the insufficient secretion of growth hormone. Growth hormone, which is mainly generated by adenohypophysis cells, can regulate the endocrine system and promote the growth of bone and muscle, thus accelerating the growth rate of the body. Therefore, it is particularly important to promote the growth and development of children with dwarfism through supplementation with exogenous growth hormone. Vitamin D is an essential nutrient for metabolism and plays an important role in the development of children. The addition of exogenous vitamin D can promote the absorption of calcium and promote bone growth and development [17, 18]. rhGH is an exogenous growth hormone preparation, which has the effect of growth hormone and can upregulate the expression of growth hormone. It can act on cells to trigger biological effects, generate GH, and combine with the GH receptors on the surface of the cell membranes to promote the proliferation of chondrocytes, stimulate the generation of osteoblasts, strengthen the differentiation and activity of osteoclasts, regulate the formation of bone collagen, and accelerate bone formation. In addition, growth and development in children are mainly achieved through two growth modes: endomembranous osteogenic growth and endochondral osteogenic growth. By supplementing exogenous vitamin D, migration and proliferation of epiphyseal plate chondrocytes and osteoblasts can be improved, and bone mineral content and bone size can be influenced, which can promote bone calcification and promote growth and development of children [19, 20].

Furthermore, IGF-1 is a peptide protein with a molecular structure similar to that of insulin. It can improve the absorption of amino acids and glucose, promote bone metabolism and synthesis, and strengthen the activity of alkaline phosphatase in osteoblasts. Growth hormone promotes the activation of vitamin D mainly through indirect or direct effects of IGF-1, so as to improve the bone mineral content, bone mineral density, and bone volume, thus promoting bone growth. Ghrelin is a brain-gut peptide that is mainly secreted by gastric mucosal cells. Its principal mechanism of action is the promotion of the secretion of growth hormone, regulation of the gastrointestinal tract, and participation in energy balance to affect growth and development. Based on the above findings, the present study statistically analyzed the expression of IGF-1 and ghrelin in children with GHD before and after treatment. The results showed that the serum IGF-1 level in the study group was higher than that in the control group, while the ghrelin level was lower than that in the control group. From the microscopic perspective of serum factors, it was further confirmed that combined treatment with rhGH and vitamin D has a high application value in GHD and can effectively regulate the serum expression of IGF-1 and ghrelin and promote the growth and development of children. In addition, there was no significant difference in the incidence of adverse reactions between the study and control groups. These results indicate that combined rhGH and vitamin D treatment for GHD not only can guarantee disease intervention but also is safe and is not associated with an increased risk of adverse reactions. In addition, during the intervention period of this study, one case of elevated fasting blood glucose development occurred in the control group, because growth hormone can promote the increase of blood glucose, while vitamin D is conducive to the control of blood glucose, and the specific mechanism is not clear.

## 5. Conclusion

In conclusion, treatment with combined rhGH and vitamin D can effectively promote the growth and development of children with GHD. It can improve bone metabolism and regulate the levels of IGF-1 and ghrelin and is a safe treatment that is worth promoting in children with GHD.

## Figures and Tables

**Table 1:** Comparison of growth and development between the two groups.

Time	Group	No. of cases	Bone age (years old)	Growth rate (cm/year)	Height (cm)
Before the treatment	Study group	70	5.69 ± 1.91	4.01 ± 0.35	101.76 ± 22.19
	Control group	30	6.02 ± 2.04	3.98 ± 0.38	103.11 ± 20.69
	*t* value		0.776	1.404	0.284
	*P* value		0.440	0.164	0.777

After 12 months of treatment	Study group	70	9.01 ± 1.10	9.62 ± 2.38	139.81 ± 16.53
	Control group	30	9.03 ± 0.98	7.91 ± 2.11	128.64 ± 13.79
	*t* value		0.173	3.402	3.246
	*P* value		0.928	0.001	0.002

**Table 2:** Comparison of bone metabolism between the two groups.

Time	Group	No. of cases	BAP (U/L)	*β*-CTX (*μ*g/L)	OC (*μ*g/L)	PINP (*μ*g/L)
Before the treatment	Study group	70	89.67 ± 26.12	0.83 ± 0.29	59.79 ± 17.10	469.62 ± 97.73
	Control group	30	91.23 ± 28.09	0.87 ± 0.35	61.56 ± 15.53	473.68 ± 93.56
	*t* value		0.268	0.593	0.487	0.193
	*P* value		0.790	0.554	0.627	0.848

After 12 months of treatment	Study group	70	173.64 ± 44.69	0.42 ± 0.18	83.37 ± 15.32	589.97 ± 103.13
	Control group	30	132.12 ± 39.64	0.59 ± 0.20	74.29 ± 12.37	541.66 ± 94.92
	*t* value		4.405	4.185	2.868	2.197
	*P* value		0.001	0.001	0.005	0.030

**Table 3:** Comparison of IGF-1 and ghrelin levels between the two groups.

Group	No. of cases	Ghrelin		IGF-1	
		Before the treatment	After 12 months of treatment	Before the treatment	After 12 months of treatment
Study group	70	6.89 ± 0.94	4.56 ± 0.39	98.29 ± 13.19	173.05 ± 19.37
Control group	30	7.01 ± 1.10	5.38 ± 0.46	102.68 ± 15.64	151.36 ± 16.62
*t* value		0.555	9.122	1.441	5.344
*P* value		0.580	0.001	0.153	0.001

**Table 4:** Comparison of adverse reactions between the two groups *n*.

Group	No. of cases	Elevated fasting blood glucose	Thyroid dysfunction	Disgusting vomits	Headache	Total incidence
Study	70	0 (0.00)	0 (0.00)	1 (1.43)	1 (1.43)	2 (2.86)
Control	30	1 (3.33)	1 (3.33)	1 (3.33)	0 (0.00)	3 (9.99)
*χ* ^2^ value						1.003
*P* value						0.317

## Data Availability

Data was included in the manuscript.
